# A Net Meta-Analysis of the Effectiveness of Different Types of Dressings in the Treatment of Diabetic Foot

This article has been retracted.

**DOI:** 10.1155/2022/4915402

**Published:** 2022-07-18

**Authors:** Ying Wang, Nan Chao, Doudou Yin

**Affiliations:** Internal Medicine, Changzhou Medical District, No. 904 Hospital the Joint Logistics Support Force of the Chinese People's Liberation Army, 213000, China

## Abstract

**Objective:**

This is an analysis of the impact of a new dressing commonly used to treat diabetic foot (DFU).

**Methods:**

Chinese and English databases were searched to collect clinical randomized controlled studies (RCTs) of various types of dressings for the treatment of DFU, and the healing rates of the different dressings were combined by reticulation meta-analysis.

**Results:**

The aggregate of the 36 RCTs included in this study analysed the healing rates of nine dressings: conventional dressing, alginate dressing, chitosan dressing, hyaluronic acid dressing, platelet-rich plasma dressing, amniotic membrane dressing, honey dressing, human recombinant growth factor dressing, and silver ionomer dressing.

**Conclusion:**

Hyaluronic acid dressing, amniotic membrane dressing, honey dressing, and platelet-rich plasma dressing are the ideal materials for topical treatment of DFU.

## 1. Introduction

Diabetic foot (DFU) is one of the common complications of diabetic patients, with a prevalence of 4% to 10% in the diabetic population [1]. DFU is caused by vascular and neuropathy of the distal lower extremity, mainly manifested as foot ulcers and deep tissue destruction. In severe cases, amputation is required, which is an important cause of disability in diabetic patients [2, 3]. Studies have shown that the risk of amputation in DFU patients is 10-30 times that of the general population, resulting in a heavy disease burden. Early prevention and aggressive treatment can reduce DFU classification and the risk of amputation [4]. Various dressings are required for local treatment of DFU, whether conventional dressings or dressings made of new synthetic materials in recent years, which can promote ulcer healing and reduce infection [5].

Diabetes foot is a kind of destructive lesion of foot or lower limb tissue in patients with diabetes. It plays a very important role in the occurrence of vascular disease, neuropathy, and infection of diabetes. In fact, vascular diseases include the diseases of large blood vessels in the lower limbs. It also includes the pathological changes of microvessels that supply nutritional nerves. In addition, many patients also have bacterial infection or other fungal infection. These three factors are all important factors leading to diabetes foot. The harm of diabetes foot is amputation, which seriously affects the quality of life of patients. In addition, the occurrence of diabetes foot actually represents that the patients' systemic vascular disease is very serious, and the survival time of patients with diabetes foot is actually greatly reduced.

With the development of biotechnology, a variety of new dressings have been clinically applied in recent years, such as amniotic membrane dressings and platelet-rich plasma dressings. The selection of appropriate dressings has positive significance for improving the therapeutic effect of DFU, reducing exudation and infection, and reducing the incidence of complications. This article intends to compare the effects of dressings commonly used in clinical treatment of DFU through a network meta-analysis, so as to provide a basis for the selection of dressings for DFU treatment.

## 2. Materials and Methods

### 2.1. Literature Inclusion Criteria

Research design: a randomized controlled clinical study (RCT) of different dressings in the treatment of DFU. (2) Study subjects: DFU patients, diabetes type 1 or 2, and Wagner grades 1-5. (3) Intervention measures: the experimental group used unconventional dressings, including alginate dressing, chitosan dressing, HA dressing, PRP dressing, amniotic membrane dressing (dHACM dressing), honey dressing (honey dressing), human recombinant growth factor dressing (hrEGF dressing), and silver ion dressing (silver ion dressing); the control group used conventional dressing (conventional dressing) or other dressings, conventional dressings including no fungal gauze, saline-soaked gauze, iodophor or povidone-iodine dressings, antibacterial dressings. (4) Outcome measures were reported: healing rate.

### 2.2. Literature Exclusion Criteria

(1) Repeated reports for the same study population, in which case the literature with the largest sample size was included; (2) the composition of the dressing was unclear, or different types of dressings were used in combination; (3) the data were incomplete; (4) literature published in languages other than Chinese and English; (5) full text cannot be obtained; (6) animal experiments and case reports.

### 2.3. Literature Search Strategy

Search Chinese and English electronic databases, Chinese databases include CNKI, Wanfang Database, and VIP database, and English databases include PubMed, Web of Science, Embase, SinoMed, and Cochrane Library. The search period was from January 2006 to December 2021. Chinese keywords: diabetic foot; dressing; bandage; randomized experiment. English search terms: diabetic foot ulcer; dressing; bandage; randomised. Search MseSH-related terms, subject headings, and free-word associations.

### 2.4. Data Extraction

Two researchers independently screened the literature, extracted data from the included literature, and consulted a third party when the two researchers had disagreements. A data collection form was developed, and the extracted data included authors, publication year, sample size, intervention program, follow-up time, and healing rate.

### 2.5. Literature Quality Evaluation

The modified Jadad scale was used to evaluate literature quality, including random sequence generation, allocation concealment, blinding, and withdrawal, with a maximum score of 7 points; ≥4 points were judged as high-quality literature [6].

## 3. Results

### 3.1. Literature Screening Process and Basic Characteristics of Included Literature

A total of 36 papers were included in this study, and the literature screening process is shown in Figure 1. Eight papers were in Chinese and 28 in English; 1541 cases were accumulated in the trial group (group T) and 1401 cases in the control group (group C). The study by Guo et al. [26] reported the effect of both honey dressing and silver ionomer dressing versus conventional dressing, and the rest were comparisons of both dressings. The follow-up period ranged from 4 weeks to 6 months, with 12 weeks being the most common. 23 publications with Jadad scores of 2-7 and ≥4 were available, representing 63.9% of the high-quality literature. The basic characteristics of the literature are shown in Table 1.

### 3.2. Meta-Analysis Results

#### 3.2.1. Evidence Network of Healing Rates

The healing rates of the 9 dressings were compared in this analysis, and the net relationship between the healing rates of different dressings is shown in Figure 2. The size of the dots in the figure represents the number of studies for that dressing, and the thickness of the line represents the number of studies comparing the 2 dressings, from which it can be seen that other dressings were most commonly compared with conventional dressings in this analysis, and the top three comparisons between the two were silver ionomer dressing and conventional dressing, PRP dressing and conventional dressing, and honey dressing and conventional dressing.

#### 3.2.2. Consistency Results

Nodal analysis showed no significant difference between direct and indirect comparisons of ulcer healing rates (*P* > 0.05), which could be analysed using a consistency model. See Table 2.

#### 3.2.3. Meta-Analysis of the Healing Rate of Different Types of Dressings

The results of the meta-analysis of the healing rate of different types of dressings are shown in Figure 3. It can be seen from Figure 3 that the healing rate of chitosan dressing, hyaluronic acid dressing, platelet-rich plasma dressing, amniotic membrane dressing, honey dressing, epidermal growth factor dressing, and silver ion dressing was significantly higher than that of conventional dressing (*P* < 0.05), while the rest of the two comparisons were not statistically different (*P* > 0.05).

#### 3.2.4. Probability Ranking and Ranking of Results

The probability ranking of different types of dressings is shown in Table 3, the highest probability of healing rate was for hyaluronic acid dressing with 50.7%, the second highest probability was for amniotic membrane dressing with 24.1%, the third highest probability was for platelet-rich plasma dressing with 17.5%, and the worst probability of healing rate was for conventional dressing with 91.6%. The results of the SUCRA ranking are shown in Table 4; the greater the SUCRA, the higher the healing rate, in order of hyaluronic acid dressing > amniotic membrane dressing > honey dressing > platelet‐rich plasma dressing > epidermal growth factor dressing > silver ion dressing > chitosan dressing > alginate dressing > conventional dressing.

As shown in Figure 4, the formula of cross-sectional survey sample size is *n* = *t*_*a*_^2^*PQ*/*d*^2^; *n* is the sample size, *P* is the prevalence of myocardial infarction, *Q* = 1 − *P*, *d* is the allowable error, *a* = 0.05, and *t*_*a*_ = 1.96. The minimum sample size is 200 cases, and the actual sample size of 280 cases of myocardial infarction was included in this study. 13 cases were dropped due to transfer and moving cases, and the rest were divided into the emergency group and the elective group of 140 cases each. Baseline information such as gender, age, and other information of patients in both groups had no effect on this study. The selected patients were all patients with myocardial infarction, and there were no shedders or dropouts at 3 months of follow-up.

Patients in both groups underwent MRI at 7-10 d and 3 months after myocardial infarction with a Philips Intera 1.5TMas-tr superconducting magnetic resonance imaging machine, with the patient in the supine position, using a chest lead cardiac gating technique and a respiratory monitoring device, and a fast breath-hold sequence scan to complete long-axis (four-chamber) and short-axis (two-chamber) cardiac cine MRI acquisition. The morphological structure of the heart was observed at the short-axis level using a fast spin-echo sequence.

### 3.3. Publication Bias

The funnel plot is shown in Figure 5 and the distribution across studies is generally symmetrical, suggesting that there is no significant publication bias.

## 4. Discussion

This study compared the effects of 9 medical dressings commonly used in clinical treatment of DFU. The results showed that 7 dressings (chitosan dressing, hyaluronic acid dressing, platelet-rich plasma dressing, amniotic membrane dressing, honey dressing, epidermal growth factor dressing, and silver ionic dressings) are more effective than conventional dressings and can achieve higher healing rates. Among the above-mentioned new dressings, hyaluronic acid dressings, amniotic membrane dressings, honey dressings, and platelet-rich plasma dressings can achieve relatively high healing rates and can be preferred.

Hyaluronic acid (HA) is a linear polymer polysaccharide composed of glucuronic acid-N-acetylglucosamine as a disaccharide unit. It is widely present in the cytoplasm and has good biocompatibility [42]. HA is one of the main components of the extracellular matrix, which plays an important role in promoting the formation of blood clots, angiogenesis, proliferation and migration of fibroblasts, regeneration of granulation tissue, and other biological processes after the occurrence of wounds or ulcers in the human body [42, 43] and can play a role in moisturizing, promoting wound healing, and regulating immune inflammatory response. Therefore, exogenous HA supplementation has a high application value in the treatment of DFU. Wound healing is a complex process, which is a process of remodeling the matrix by a variety of cells and their products, and different cells need to move in orderly. Studies have shown that in the early stage of wound healing, cells secrete a large amount of HA, which can promote wound contraction, increase the activity of neutrophils, and accelerate their phagocytosis of necrotic tissues and bacteria; the molecular fragments generated after the degradation of macromolecular HA can stimulate blood vessels, generated and involved in subsequent reconstructions [44]. HA can also induce cell aggregation and promote the formation of blood vessels within the collagen and fibrin matrix, thereby promoting wound healing [45]. This study shows that the treatment effect of HA dressing on DFU is better than that of conventional dressing, which can achieve a better healing rate, and the healing rate ranks first, indicating that it has high applicability in the treatment of DFU and can be used as a local treatment for DFU, one of the preferred options.

Amniotic membrane is a new type of topical material for ulcers, which maintains moistening of the wound, reduces exudation, and inhibits microbial colonization. Amniotic membranes are rich in growth factors and collagen and have effects such as inducing epithelial regeneration, which can promote wound repair and tissue regeneration [46]. In recent years, commercialised amniotic membrane products have increased in clinical use and have shown good results in the treatment of difficult ulcers such as DFU. A study by Litwinuk et al. [47] showed that amniotic membrane contains high levels of metalloproteinase (MMP) inhibitors, which inhibit MMP-2 and MMP-9 activity associated with chronic refractory wounds, thereby promoting wound healing [47]. The treatment of DFU with amniotic dressings has been supported by several clinical studies in recent years, with an efficiency rate of over 90% [29, 48, 50]. The weak acidity of honey can also inhibit the growth of pathogenic bacteria, thereby exerting debridement and anti-infection effects. In addition to the above effects, honey also has a strong ability to promote healing. It can activate macrophages, promote the transition of wounds from chronic inflammation to proliferation and reconstruction, promote the division of B lymphocytes and T lymphocytes, and increase neutrophil cellular activity, thereby accelerating the repair process [51–54]. In addition, PRP contains a large amount of fibrin, which can provide a biological scaffold for cells in the repair process and promote wound shrinkage [15, 28]. PRP also has a strong anti-infective effect, which can inhibit the colonization and growth of common skin infection pathogens such as Staphylococcus aureus and reduce the risk of local infection [15]. This study shows that the healing rate of PRP dressing ranks fourth, and its therapeutic effect on DFU is significantly better than that of conventional dressings.

In conclusion, hyaluronic acid dressings, amniotic membrane dressings, honey dressings, and platelet-rich plasma dressings are ideal materials for local treatment of DFU and can be preferred. However, this study has certain limitations, which are mainly reflected in the following aspects: only Chinese and English literatures are included, and the representativeness may be insufficient; some literatures are of low quality, which may affect the strength of the evidence; this analysis only considers the main effect of healing rate indicators, and economic benefits are not explored.

## Figures and Tables

**Figure 1:** Literature screening process.

**Figure 2:** Network diagram of healing rate.

**Figure 3:** Results of reticulated meta-analysis of healing rates for different types of dressings. Notes: Con: conventional dressing; Alg: alginate dressing; Chi: chitosan dressing; Ha: HA dressing; Prp: PRP dressing; Hacm: dHACM dressing; Hon: honey dressing; Egf: hrEGF dressing; Sil: silver ion dressing.

**Figure 4:** SUCRA diagram for different types of dressings.

**Figure 5:** Funnel diagram. Notes: A: conventional dressing; B: alginate dressing; C: chitosan dressing; D: HA dressing; E: PRP dressing; F: dHACM dressing; G: honey dressing; H: hrEGF dressing; I: silver ion dressing.

**Table 1:** Basic characteristics of the included literature.

Author	Year	DFU grading	Sample size (T/C)	Intervention programs		Follow-up visit time	Jadad
				T	C		
Kamaratos [7]	2012	1~2 level	32/31	Honey dressing	Conventional dressing	16 weeks	5
Driver [8]	2006	—	19/21	PRP dressing	Conventional dressing	12 weeks	4
Jude [9]	2007	1~2 level	65/65	Silver ion dressing	Alginate dressing	8 weeks	5
Imran [10]	2015	1~2 level	179/169	Honey dressing	Conventional dressing	120 d	4
Mohajeri-Tehrani [11]	2016	2~4 level	27/30	dHACM dressing	Conventional dressing	6 weeks	5
Jan [12]	2012	1~4 level	50/50	Honey dressing	Conventional dressing	10 weeks	4
Park [13]	2019	1~2 level	17/13	Chitosan dressing	Conventional dressing	12 weeks	7
Lee [14]	2016	1~2 level	13/12	HA dressing	Conventional dressing	12 weeks	7
Elsaid [15]	2019	—	12/12	PRP dressing	Conventional dressing	20 weeks	5
Lobmann [16]	2020	1~2 level	126/114	Alginate dressing	Conventional dressing	20 weeks	4
Ahmed [17]	2016	—	28/28	PRP dressing	Conventional dressing	—	3
Jung [18]	2016	1~2 level	137/71	Chitosan dressing	Conventional dressing	12 weeks	5
Gude [19]	2017	1~4 level	66/63	PRP dressing	Conventional dressing	12 weeks	6
You [20]	2014	1~2 level	31/32	HA dressing	Conventional dressing	12 weeks	5
Essa [21]	2021	1~2 level	40/40	Silver ion dressing	Conventional dressing	12 weeks	4
Malligurki [22]	2021	1~2 level	25/25	Silver ion dressing	Conventional dressing	8 weeks	3
Zeleníková [23]	2019	—	20/20	Honey dressing	Conventional dressing	90 d	3
Chen [24]	2020	1~2 level	30/30	Alginate dressing	Conventional dressing	—	3
Lu [25]	2012	1~3 level	45/34	Silver ion dressing	Conventional dressing	—	2
Guo [26]	2013	2~3 level	36/37	Honey dressing	Conventional dressing	—	2
Guo [26]	2013	2~3 level	37/37	Silver ion dressing	Conventional dressing	—	2
Viswanathan [27]	2020	1~2 level	27/23	hrEGF dressing	Conventional dressing	30 d	4
Elsaid [15]	2020	1~3 level	12/12	PRP dressing	Conventional dressing	20 weeks	5
Xie [28]	2020	1~4 level	25/23	PRP dressing	Conventional dressing	4 weeks	4
Tettelbach [29]	2019	—	54/56	dHACM dressing	Alginate dressing	12 weeks	7
Fu [30]	2018	2~3 level	32/32	PRP dressing	Alginate dressing	8 weeks	3
Park [31]	2018	1~2 level	82/85	hrEGF dressing	Conventional dressing	12 weeks	7
Gupta [32]	2018	—	15/15	Silver ion dressing	Conventional dressing	8 weeks	4
Liu [33]	2021	—	70/70	Silver ion dressing	Conventional dressing	4 weeks	3
He [34]	2016	—	40/40	Silver ion dressing	Conventional dressing	—	3
Agarwal [35]	2015	2~3 level	30/30	Silver ion dressing	Conventional dressing	8 weeks	4
Wu [36]	2014	1~3 level	22/23	hrEGF dressing	Conventional dressing	12 weeks	3
Gomez-Villa [37]	2014	1~2 level	17/17	hrEGF dressing	Conventional dressing	8 weeks	5
Zelen [38]	2013	1~2 level	13/12	dHACM dressing	Conventional dressing	6 weeks	4
Eldeen [39]	2012	—	20/20	Honey dressing	Alginate dressing	6 months	3
Ma [40]	2012	1~2 level	20/20	dHACM dressing	Conventional dressing	—	3
Liu [41]	2006	1~5 level	27/26	hrEGF dressing	Conventional dressing	—	3

**Table 2:** Agreement between direct and indirect comparisons of nodal analysis of healing rates for different types of dressings.

Comparison group	Direct comparison		Indirect comparison		*P*
	OR	SD	OR	SD	
A vs. B	1.957	0.693	1.916	0.918	0.884
A vs. C	1.379	0.816	1.167	1.221	0.885
A vs. E	1.303	0.546	2.352	1.249	0.442
A vs. F	1.812	0.763	1.694	1.204	1.428
A vs. G	1.192	0.600	2.188	0.950	0.374
A vs. I	1.156	0.410	2.383	1.890	0.289
B vs. E	1.341	1.128	0.292	0.766	0.442
B vs. F	0.865	1.074	0.983	0.941	0.934
B vs. G	2.539	1.470	0.150	0.724	0.145
B vs. I	1.079	1.085	0.209	0.682	0.497
C vs. G	0.281	1.086	0.068	0.987	0.885
G vs. I	0.770	1.326	-0.435	0.698	0.423

Notes: A: conventional dressing; B: alginate dressing; C: chitosan dressing; D: HA dressing; E: PRP dressing; F: dHACM dressing; G: honey dressing; H: hrEGF dressing; I: silver ion dressing.

**Table 3:** Probability ranking of healing rates (%).

Sort by	Con	Alg	Chi	Ha	Prp	Hacm	Hon	Egf	Sil
Best	0.0	0.3	6.9	50.7	7.0	21.4	7.0	4.6	2.1
2^nd^	0.0	1.2	11.7	16.1	14.8	24.1	13.9	10.7	7.5
3^rd^	0.0	2.9	12.2	8.2	17.5	15.2	17.4	13.5	13.0
4^th^	0.0	5.3	11.9	6.5	16.1	12.1	17.0	14.3	16.9
5^th^	0.0	8.9	12.4	5.5	15.2	9.4	15.8	13.9	19.0
6^th^	0.0	14.9	12.2	4.4	12.3	7.5	13.8	14.7	20.1
7^th^	0.0	23.4	15.2	4.4	10.8	6.6	10.2	14.8	14.4
8^th^	8.2	38.9	15.4	3.7	6.2	3.3	4.7	12.8	6.9
Worst	91.6	4.3	2.2	0.6	0.1	0.3	0.1	0.7	0.0

Notes: Con: conventional dressing; Alg: alginate dressing; Chi: chitosan dressing; Ha: HA dressing; Prp: PRP dressing; Hacm: dHACM dressing; Hon: honey dressing; EGF: hrEGF dressing; Sil: silver ion dressing.

**Table 4:** SUCRA ranking of different dressing healing rates.

Type of dressing	SUCRA	Probability of the highest healing rate (%)	Average sorting
Ha	80.9	50.7	2.5
Hacm	71.1	21.4	3.3
Hon	59.1	7.0	4.3
Prp	58.8	7.0	4.3
EGF	50.8	4.6	4.9
Sil	50.5	2.1	5.0
Chi	50.2	6.9	5.0
Alg	27.5	0.3	6.8
Con	1.1	0.0	8.9

Notes: Con: conventional dressing; Alg: alginate dressing; Chi: chitosan dressing; Ha: HA dressing; Prp: PRP dressing; Hacm: dHACM dressing; Hon: honey dressing; EGF: hrEGF dressing; Sil: silver ion dressing.

## Data Availability

The experimental data used to support the findings of this study are available from the corresponding author upon request.
